The article "Effect of High-Quality Nursing Based on Comprehensive Nursing on the Postoperative Quality of Life and Satisfaction of Patients with Malignant Glioma" was retracted in 2023. Reasons: suspected computer-generated content; unreliable results or conclusions; concerns about the data; concerns about the results or conclusions.

# Effect of High-Quality Nursing Based on Comprehensive Nursing on the Postoperative Quality of Life and Satisfaction of Patients with Malignant Glioma

**DOI:** 10.1155/2022/9345099

**Published:** 2022-04-27

**Authors:** Xue Gong, Wei Wu, Dengyu Xing, Xu Guo, Meng Yang

**Affiliations:** ^1^The Sixth Department of Neurosurgery, First Affiliated Hospital of Harbin Medical University, Harbin, Heilongjiang, China; ^2^Emergency Department, Harbin Traditional Chinese Medicine Hospital, Harbin, Heilongjiang, China; ^3^Emergency Medical Ward, First Affiliated Hospital of Harbin Medical University, Harbin, Heilongjiang, China

## Abstract

**Objective:**

To explore the effect of high-quality nursing based on comprehensive nursing on postoperative quality of life and satisfaction of patients with malignant glioma.

**Methods:**

From September 2017 to May 2020, 86 patients with malignant glioma treated in our hospital were recruited and assigned (1 : 1) to receive either comprehensive nursing (comprehensive group) or high-quality nursing plus comprehensive nursing (high-quality group). Outcome measures included preoperative and postoperative self-rating anxiety scale (SAS) scores, self-rating depression scale (SDS) scores, quality of life, and nursing satisfaction.

**Results:**

High-quality nursing plus comprehensive nursing was associated with significantly lower SAS and SDS scores versus comprehensive nursing alone (*P* < 0.05). Patients receiving high-quality nursing plus comprehensive nursing showed higher quality of life scores versus those only given comprehensive nursing (*P* < 0.05). High-quality nursing plus comprehensive nursing resulted in higher nursing satisfaction of the patients versus comprehensive nursing alone (*P* < 0.05).

**Conclusion:**

High-quality nursing can relieve the negative emotions of patients with malignant glioma and significantly enhance their quality of life, thereby improving the nursing satisfaction of patients with nursing, so it is worthy of clinical application.

## 1. Introduction

Glioma is a common clinical malignant tumor of the central system characterized by high morbidity, rapid development, and high lethality [1]. Brain gliomas are most common in people aged 40–70 years. Its symptoms include headache, dizziness, nausea, vomiting, tinnitus, and papilledema. In severe cases, epilepsy and various body dysfunctions may occur [2]. At present, surgery is one of the main methods of clinical treatment of gliomas. It can remove glial tumor cells and relieve the patient's intracranial hypertension, thereby enhancing the survival and the quality of life of patients [3]. However, the operation is invasive, which is associated with damages to the functional area of the body and complications, thus compromising the prognosis of the patient [4]. Therefore, active and effective nursing interventions are necessitated for patients postoperatively to eliminate the patients' negative emotions and improve the quality of life of patients [5]. The concept of high-quality nursing based on comprehensive nursing is to help patients improve their postoperative quality of life and psychological state, with psychological motivation for patients and encouragement of families' participation [6]. In this study, 86 patients with malignant glioma who were treated in our hospital from September 2017 to May 2020 were recruited to explore the influence of high-quality nursing on quality of life and satisfaction of patients after tumor surgery to provide a reference for clinical practice.

## 2. Materials and Methods

### 2.1. Baseline Data

From September 2017 to May 2020, 86 patients with malignant glioma treated in our hospital were recruited and assigned (1 : 1) to receive either comprehensive nursing (comprehensive group) or high-quality nursing plus comprehensive nursing (high-quality group). The research was approved by the Ethics Committee of the First Affiliated Hospital of Harbin Medical University, No. Har2971.

### 2.2. Inclusion and Exclusion Criteria

Inclusion criteria were as follows: all met the diagnostic criteria in the Guidelines for the Diagnosis and Treatment of Glioma of the Central Nervous System in China, with a diagnosis of gliomas confirmed by pathology and other examinations, patients were informed of the study and voluntarily signed the informed consent, patients received conventional craniotomy for tumor resection, and with an expected survival of ≥3 months. Exclusion criteria were as follows: patients who were unconscious, which prevented cooperation, with severe cardiovascular diseases, with severe heart, liver, kidney, and other organ diseases, and with other malignant tumors or tumors metastases.

### 2.3. Nursing Methods

Patients in both groups received three-dimensional conformal radiation therapy 2 weeks after surgical resection of the tumor. The irradiation dose was 2 Gy/time/d, 5 times/week, and the total dose did not exceed 60 Gy.

The patients in the comprehensive group were given comprehensive nursing, which included health education, vital signs-related indicators monitoring, dietary guidance, postoperative rehabilitation exercises, and discharge guidance.

The patients in the high-quality group received high-quality nursing plus comprehensive nursing. The specific methods are as follows: upon admission, the nursing staff help the patients quickly familiarize the treatment environment to facilitate their following treatment cooperation: the patients were instructed and accompanied by nursing staff in various preoperative and postoperative physical examinations to reduce their psychological pressure [7]; 1-2 days preoperatively, the patients were given operation precautions and health education to avoid perioperative stress and help them to better understand the disease and stabilize their emotions; cases with similar treatment procedures were introduced to the patients to eliminate their anxiety and fear [8]; 1 day preoperatively, the patients were given perioperative information such as operating room environment, anesthesia methods, and the general procedure of the operation; 30 minutes preoperatively, the patients were comforted when entering the operation room to help them to eliminate anxiety and fear; the preoperative preparation after anesthesia such as indwelling urinary catheter was performed to reduce the discomfort of the patient [9]; invasive operations such as venous blood collection and intravenous infusion were performed by skilled nurses after surgery; and the patients' conditions were strictly monitored to promptly resolve their issues [10].

### 2.4. Observation Indicators

1. The anxiety and depression scores of the two groups were compared. The self-rating anxiety scale (SAS) [11] was used to evaluate the anxiety of the patients, with a score of 0–100 points and a cutoff value of 50 points, in which a score of 50–59 points indicates mild anxiety, 60–69 points indicates moderate anxiety, and over 69 points indicate severe anxiety. The self-rating depression scale (SDS) was used to evaluate the depression of the patients, with a score of 0–100 points and a cutoff value of 53 points, in which a score of 53–62 points indicates mild depression, 63–72 points indicates moderate depression, and over 73 points indicates severe depression.
2. The World Health Organization Quality of Life Scale (WHOQOL-100) [12] was used to evaluate the quality of life of patients from six dimensions: physical health, psychological state, independence, social relations, personal beliefs, and relationship with the environment. The full score of each item is 100 points, and the score is positively correlated with the quality of life.
3. The nursing satisfaction of the two groups of patients was compared, and the nursing satisfaction questionnaire made by the hospital was used for evaluation. There are 20 questions, and the patients scored them according to the nursing satisfaction of the hospital, with a good reliability and validity, 5 points for each question. A total score of <70 points indicates dissatisfied, 70–89 points indicates satisfied, and ≥90 points indicates highly satisfied. Satisfaction = (highly satisfied cases + satisfied cases)/total number of cases × 100%.

### 2.5. Statistical Analysis

The data analyses were performed using SPSS 20.0. Measurement data were expressed as ($\bar{x}\pm s$), and the independent samples *t*-test was used for comparison. Enumeration data were expressed as the number of cases (rate), and the *X*^2^ test was used for comparison. Statistical significance was assumed at *P* < 0.05.

## 3. Results

### 3.1. Comparison of Baseline Data

In the comprehensive group, there were 23 males and 20 females, aged 40–68 years. There were 22 males and 21 females in the high-quality group, aged 40–70 years. There was no significant difference in general data such as gender, age, and tumor location between the two groups, as given in Table 1.

### 3.2. Comparison of SAS and SDS Scores between the Two Groups of Patients

Before nursing, there was no significant difference in the SAS and SDS scores between the two groups of patients (*P* > 0.05). High-quality nursing plus comprehensive nursing was associated with significantly lower SAS and SDS scores versus comprehensive nursing alone (*P* < 0.05, Table 2).

### 3.3. Comparison of Quality of Life Scores between the Two Groups of Patients

Before nursing, there was no significant difference in the scores of quality of life between the two groups of patients (*P* > 0.05). Patients receiving high-quality nursing plus comprehensive nursing showed higher quality of life scores versus those only given comprehensive nursing (*P* < 0.05), as given in Table 3.

### 3.4. Comparison of Nursing Satisfaction between the Two Groups of Patients

High-quality nursing plus comprehensive nursing resulted in higher nursing satisfaction of the patients versus comprehensive nursing alone (*P* < 0.05) (Table 4).

## 4. Discussion

Glioma is a common primary intracranial tumor that damages the brain tissue and leads to complications and even death, which seriously compromises the life and safety of patients [11]. Surgical resection is the mainstay of treatment for gliomas currently. However, the prognosis of patients after surgical resection of gliomas is unsatisfactory [12]. Zhang et al. [13] pointed out that in addition to active treatment for malignant glioma patients, the scientific and reasonable nursing intervention also plays a crucial role in the postoperative rehabilitation of patients. The previous comprehensive care can only meet the basic needs of patients but fails to eliminate their negative emotions, resulting in a poor prognosis [14].

Thus, high-quality nursing is essential to improving the nursing effect and clinical satisfaction [15]. Standardized nursing helps patients eliminate their negative emotions and allows patients to face treatment with a positive and optimistic attitude, preventing disease development from mitigating negative emotions [16]. The results of the present study showed that high-quality nursing plus comprehensive nursing was associated with significantly lower SAS and SDS scores versus comprehensive nursing alone, which indicates that high-quality nursing can better help patients relieve their negative emotions. The reason may be that the enhanced disease and treatment knowledge by health education lessened the patients' psychological burden [17].

Fang et al. pointed out that good postoperative nursing can effectively enhance the quality of life of patients [18]. In the present study, patients receiving high-quality nursing plus comprehensive nursing showed higher quality of life scores versus those only given comprehensive nursing, which was consistent with the relevant research results of the previous research [19]. The reason may be that high-quality nursing focuses on the overall recovery of the patient after surgery, and the strict monitoring of vital signs contributes to better understanding of the patients' condition, which contributes to the enhancement of postoperative quality of life [20]. Moreover, high-quality nursing plus comprehensive nursing resulted in higher nursing satisfaction of the patients versus comprehensive nursing alone, suggesting a good recognition of the high-quality nursing by the patients and their families [21].

N-myc downstream-regulated gene 2 (NDRG2) belongs to the NDRG family, which includes four members, NDRG1, NDRG2, NDRG3, and NDRG4. NDRG2 expression is significantly reduced or absent in many human tumor tissues, such as breast cancer, liver cancer, colorectal cancer, and malignant glioma, suggesting that NDRG2 has an inhibitory effect on tumorigenesis. NDRG2 can inhibit tumor cell proliferation through signaling pathways such as TCF/*β*-catenin and P1 K/Akt and promote apoptosis through p53 and HIF pathways. Therefore, NDRG2 is currently considered an effective oncogenic candidate molecule. However, a growing body of evidence suggests that in addition to its oncogenic effects, NDRG2 also plays an important role in normal CNS function and disease. For example, NDRG2 can promote neuronal axon growth and synapse formation and participate in the antiapoptotic mechanism of ischemic electroacupuncture preconditioning in rat brain, which can be a new molecular target for the treatment of depression and epilepsy.

In recent years, the research of Chinese medicine for the treatment of glioma has become a hotspot. The herbal medicine Yadanziyou Oleum Bruceae is used in combination with radiotherapy for the treatment of malignant glioma. Yadanziyou Oleum Bruceae is an active ingredient extracted from the mature fruits of *Brucea javanica*, which is one of the most active Chinese medicinal preparations for the treatment of tumors. The main components of its anticancer activity are oleic acid and linoleic acid, which have the dual effects of antitumor and improving the immune function of the body. It is proved that Yadanziyou Oleum Bruceae is a cell cycle nonspecific antitumor drug, which has certain killing and inhibiting effects on tumor cells in GO, G1, S, G2, and M phases, significantly inhibits the synthesis of tumor cell DNA, antiproliferation, disrupts tumor cell biofilm, enhances cellular immune function, protects bone marrow, and elevates white blood cells [9–12]. Studies have shown that 90% of Yadanziyou Oleum Bruceae with a diameter of 1 um can rapidly cross the blood-brain barrier and enter the brain and cancerous tissues. It has a good inhibitory effect on intracranial malignant tumors. Compared with commonly used chemotherapeutic drugs, it has certain advantages in improving the quality of life and prolonging the survival of patients with advanced cancer [15, 16]. The limitation of this study is the absence of an elaboration on the care of adverse effects caused by chemotherapy, which will be investigated in future studies.

## 5. Conclusion

High-quality nursing can relieve the negative emotions of patients with malignant glioma and significantly enhance their quality of life, thereby improving the nursing satisfaction of patients with nursing, so it is worthy of clinical application.

## Figures and Tables

**Table 1:** Baseline data (*n* (%)).

	Comprehensive group (*n* = 43)	High-quality group (*n* = 43)	*t*/*x*^2^	*P*
Gender			0.047	0.829
Male	23	22		
Female	20	21		
Mean age (year)	51.24 ± 5.72	51.46 ± 5.63	−0.18	0.858
Tumor site			0.191	0.662
Supratentorial glioma	26	24		
Pontine glioma	17	19		

**Table 2:** Comparison of anxiety (SAS) and depression (SDS) scores between the two groups of patients (*x* ± *s*).

Groups	*n*	SAS (point)		SDS (point)	
		Before nursing	After nursing	Before nursing	After nursing
Comprehensive group	43	44.58 ± 3.36	37.63 ± 2.57	43.34 ± 3.21	39.42 ± 5.78
High-quality group	43	44.69 ± 3.29	28.33 ± 2.97	43.40 ± 3.25	28.97 ± 5.21
*T*	—	−0.153	15.527	−0.086	8.806
*P*	—	0.879	＜0.001	0.932	＜0.001

**Table 3:** Comparison of quality of life scores between the two groups of patients (*x* ± *s*).

Groups	*n*	Physical health		Mental state		Independence ability		Social relationship		Personal beliefs		Relationship with the surrounding environment	
		Before nursing	After nursing	Before nursing	After nursing	Before nursing	After nursing	Before nursing	After nursing	Before nursing	After nursing	Before nursing	After nursing
Comprehensive group	43	60.34 ± 5.72	76.12 ± 9.34	57.28 ± 4.16	70.42 ± 6.18	50.27 ± 2.87	68.74 ± 5.22	60.11 ± 4.35	72.49 ± 7.65	65.74 ± 9.21	75.26 ± 8.58	62.57 ± 6.35	70.52 ± 4.29
High-quality group	43	60.53 ± 5.56	84.58 ± 8.97	57.50 ± 4.25	80.61 ± 5.29	50.13 ± 2.69	80.43 ± 3.42	60.20 ± 4.18	82.13 ± 5.97	65.59 ± 9.15	83.42 ± 7.93	62.70 ± 6.42	81.48 ± 5.13
*T*	—	−0.156	−4.284	−0.243	−8.214	0.233	−12.284	−0.098	−6.514	0.076	−4.58	−0.094	−10.747
*P*	—	0.876	＜0.001	0.809	＜0.001	0.816	＜0.001	0.922	＜0.001	0.94	＜0.001	0.925	＜0.001

**Table 4:** Satisfaction (*n* (%)).

Groups	*n*	Dissatisfied	Satisfied	Very satisfied	Total
Comprehensive group	43	15	16	12	28 (65%)
High-quality group	43	3	15	25	40 (93%)
*T*	—	—	—	—	10.118
*P*	—	—	—	—	0.001

## Data Availability

No data were used to support this study.
